# Mentalized affectivity in a nutshell: Validation of the Italian version of the Brief-Mentalized Affectivity Scale (B-MAS)

**DOI:** 10.1371/journal.pone.0260678

**Published:** 2021-12-02

**Authors:** Marianna Liotti, Grazia Fernanda Spitoni, Vittorio Lingiardi, Antonella Marchetti, Anna Maria Speranza, Annalisa Valle, Elliot Jurist, Guido Giovanardi

**Affiliations:** 1 Department of Dynamic, Clinical and Health Psychology, Sapienza University of Rome, Rome, Italy; 2 Research Unit on Theory of Mind, Department of Psychology, Università Cattolica del Sacro Cuore, Milan, Italy; 3 Clinical Psychology at the City College of New York, and The Graduate Center of the City University of New York, New York, New York, United States of America; Universita Cattolica del Sacro Cuore Sede di Roma, ITALY

## Abstract

The term “mentalized affectivity” describes the ability to reflect on, process, modulate and express emotions through the prism of autobiographical memory. It represents a bridge concept that integrates previous contributions on emotion regulation and mentalization, offering a quite unique perspective on affective and reflective functioning. The overall aim of this study was to validate the Brief-Mentalized Affectivity Scale (B-MAS), a 12-items self-report instrument, on the Italian population. We tested both the factorial validity of the instrument and its reliability and convergent validity with other similar constructs. We also obtained normative data for the Italian population, broken down by gender. Participants (n = 389) were recruited through snowball sampling. Data was collected through an online survey. Besides the Brief-Mentalized Affectivity Scale, the survey included an ad hoc schedule with questions investigating socio-demographic characteristics, and self-report measures of empathy and reflective functioning. Statistical analysis has shown a three-component (Identifying, Processing, and Expressing emotions) hierarchical structure underlying mentalized affectivity, mirroring the model already proposed in the original validation of the instrument. Moreover, the B-MAS showed good psychometric properties for what regards both reliability and convergent validity. The results of our study highlight the good operationalization and robust empirical foundation of the construct, revealing that the B-MAS is a promising instrument to assess mentalized affectivity. Its brevity makes it particularly valuable both in clinical and research contexts, and the normative data provided in this study will allow an easy comparison with the scores obtained by other samples (clinical and non-clinical).

## Introduction

### Mentalization

The concept of mentalization, developed by Fonagy and colleagues [1–3], has been one of the most fruitful over recent years, both in research and clinical practice. Bateman and Fonagy [4, p. xxi] define it as “The mental process by which an individual implicitly and explicitly interprets the actions of oneself and others as meaningful on the basis of intentional mental states such as personal desires, needs, feelings, beliefs, and reasons”. This concept brings together many past theoretical formulations: from ego psychology to object relations theory and, most notably, attachment theory [5].

Over time, however, Fonagy and colleagues’ notion of mentalization (or *reflective functioning*) has evolved. At first, much emphasis was given to mentalization as an ability that emerges from early experiences with caregivers and may thus be impaired by a traumatic attachment or other adverse experiences. Recently, however, the concept has been broadened to encompass other psychological processes and notions, such as social learning and epistemic trust (an expression which refers to the inclination to appraise new, socially transmitted information as trustworthy, useful, and personally relevant [6–8]). Different aspects of mentalization have emerged: implicit or explicit, automatic or voluntary, regarding self or others, cognitive or affective [9–11]. Such expansion, even though valuable for clinical understandings, has brought to light how the many facets of mentalization overlaps with other concepts [12, 13].

### Mentalized affectivity

Concerning affective mentalization more specifically, Elliot Jurist [10, 14–16] has proposed the notion of *mentalized affectivity*, defined as “the capacity to reflect on emotions in light of autobiographical memory” [10, p. ix]. Its source lies in “the desire to understand how one’s past and identity inform one’s emotional experience” [10, p. 3], and it is influenced by beliefs, values, cognitive processes, personality patterns, and life experiences. According to Jurist [10], this aspect of mentalization is the most relevant for psychotherapy: not only it connects much of what we know about emotional recognition, expression, and regulation, but it also emphasizes various fundamental aspects of our psychological wellbeing—such as empathy, curiosity, cognitive flexibility, and love for truth. Furthermore, fostering our mentalized affectivity means promoting our ability to develop new and more adaptive perspectives on ourselves. The ability to mentalize is directly connected to affective regulation, which does not depend only on the capacity to modulate and express emotions but also to re-evaluate their meaning in the light of our present and past experiences.

As already noted, however, being able to operationalize and empirically measure this concept appears vital. To do this, Jurist and colleagues have developed a self-report instrument called Mentalized Affectivity Scale (MAS; [17]). In addition, the authors have recently validated a shorter version of the tool, the Brief-Mentalized Affectivity Scale (B-MAS; [18]). We will further illustrate both the long- and short- form of the instrument in the next paragraph.

### Mentalized Affectivity Scale (long and brief form) and its relationship with other measures

The instrument was designed to assess individuals’ mentalized affectivity (and its potential development over time), extending the field of self-report measures of emotion regulation. Indeed, various instruments can be utilised to evaluate individuals’ ability to recognize, regulate and express emotion. The Emotion Regulation Questionnaire (ERQ; [19]), the Empathy Quotient (EQ; [20]), the Difficulties in Emotion Regulation Scale (DERS; [21]), and the Toronto Alexithymia Scale (TAS-20; [22]) are just some examples. However, none of these tools assess all three elements of our emotional functioning together.

Furthermore, none of the instruments cited above evaluates how our ability to reflect on our past and present experiences can affect our ability to identify, modulate and communicate to others our feelings and welcome them as part of our identity [10]. Being a bridge concept between mentalization and affective regulation—and focusing the attention on the interrelatedness between emotions, memory, and life experiences—the MAS represents a new and original instrument in psychological literature. It has already been translated into many languages, such as Korean, Japanese, Taiwanese, Mandarin, German, Spanish, Persian, Turkish, Bulgarian, Russian, and Italian (https://www.mentalizedaffectivity.net/scale).

In its long-form version, the MAS consists of 60 items. The initial validation of the instrument [17] has revealed a solid three-component structure underlying mentalized affectivity. Such factors, which reflect the three elements postulated theoretically by Jurist [10], are 1) Identifying emotions, 2) Processing emotions, and 3) Expressing emotions. Identifying emotions refers not only to the ability to be aware and correctly identify and label one’s feelings but also to reflect on the elements that influence them; it has to do with curiosity and openness. Processing emotions involves the ability to regulate them, modulating their intensity or extent through mechanisms such as cognitive reappraisal. Finally, Expressing emotions refers to the ability to communicate them and convey their meaning, both inwardly and outwardly. All three of these factors are interconnected, and all of them are related to one’s sense of agency.

The Italian validation of the MAS has found a five-factor hierarchical structure [23]. These are Identifying Emotions, Expressing Emotions, Curiosity about Emotions, Processing Emotions, and Autobiographical Memory.

The MAS possesses good psychometric properties [17, 23]. However, since it consists of 60 items (35 in the Italian version), its length may make it too demanding to be used in clinical and research settings. Greenberg and colleagues [18] have thus developed the Brief-Mentalized Affectivity Scale (B-MAS) to create a less burdensome tool still able to capture all three components of the original one. After selecting 12 representative items among the original 60, the authors asked various mentalization and emotion regulation experts to evaluate if the chosen items (grouped in three main clusters) appropriately measured each of the three original factors. The results confirm that the B-MAS is a valid and useful measure of emotion regulation and mentalization, with excellent psychometrical properties. It shows the same three-component structure of the long-form scale. Furthermore, it possesses strong construct validity with other more notorious scales for emotion regulation, such as the ERQ, the DERS, and the TAS-20, as well as with the Reflective Functioning Questionnaire (RFQ; [24])–while offering new perspectives within the emotion regulation and mentalization context.

Moreover, Greenberg and colleagues [18] also investigated the correlation between mentalized affectivity and other dimensions of psychological functioning in a clinical population. They found that the scores obtained at the B-MAS were predictive of numerous mental health diagnoses, and of the general degree of wellbeing (and more so than traditional measures). The B-MAS seems thus to represent a valuable tool in clinical settings, thanks to its brevity and ease of administration and scoring.

### Aims of the present study: Italian validation of the B-MAS

The overall aim of the present research was to validate the brief measure of mentalized affectivity in a cohort of Italian adults. Towards that end, we aimed to (1) test the factorial structure of the instrument (via Exploratory Factor Analysis with Promax rotation—EFA and Confirmatory Factor Analysis—CFA); (2) test the instrument reliability and convergent validity by examining the associations between mentalized affectivity and empathy (tested with the Empathy Quotient), as well as mentalized affectivity and reflective functioning (tested with the Reflective Functioning Questionnaire); and (3) study the effect of Demographics and obtain Normative data.

## Methods

### Participants

A total of 389 participants completed the study. Of those, 189 (47%) were male, 192 (49%) were female, 17 (4%) were non-binary. Participants’ age ranged from 18 and 65 years, with a mean of 27.30 (*SD* = 8.99). All participants were Italian. The majority (N = 167, 43%) of respondents reported having completed high school, whereas 86 (22%) completed a bachelor’s degree, 86 (22%) had a master’s degree, and 28 (7%) had a Ph.D. Only 3 (0.8%) reported a primary school educational level. Nineteen (5%) subjects did not give any information about their educational level.

### Procedure

The study was conducted through an online survey, recruiting participants via several professional mailing lists and social media. It took circa 30–40 minutes to be completed. Participants took the survey using the platform SurveyMonkey. Responses were anonymous, and participants could stop at any time and restart later or decide to withdraw from the study without any penalty. They were also informed that it was possible to contact the principal investigator of the study before, during, or after their participation to ask for any clarification.

The survey has been online from January 05 to April 12, 2021. As mentioned above, participants were recruited through snowball sampling (e.g., via email invitation and dissemination through social media channels such as Facebook and Instagram). Respondent’s IP addresses were logged to prevent duplicate answers. Only participants who responded to all the questions were included in the study. Inclusion criteria were being aged 18 years or older and speaking Italian. The study was approved by the local Ethics Committee.

### Measures

The survey included an ad-hoc questionnaire to collect information on socio-demographic variables, a shorter version of the Empathy Quotient (EQ; [20]), and the Reflective Functioning Questionnaire (RFQ; [24]). Each measure will be described more in detail below. The 12 items of the B-MAS instrument were translated by the authors and then back-translated into English by an independent translator with no knowledge of the instrument. We then revised some minor expressions to achieve better quality and accuracy.

#### Socio-demographic variables

Participants were asked to complete a socio-demographic questionnaire to collect information on their biological sex, gender, nationality, age, and level of education.

#### Convergent validity: Correlations with empathy and reflective functioning levels

Empathy and reflective functioning were chosen as the two more significant constructs for convergent validity for the following reasons. Empathy, defined as the ability to understand others’ thoughts and feelings and to predict their behaviour based on that information [20], is a concept strictly related to mentalized affectivity. Indeed, to predict other’s emotional responses, we have to elicit and utilise our past and present internal affective representations—and the more individuals use such representations when attempting to understand the emotional reactions of others, the higher their levels of empathy are [25]. Following Rinaldi and colleagues [23], we also correlated the B-MAS subscales to RFQ subscales (Certainty, RFQ_C, and Uncertainty, RFQ_U). Since reflective functioning represents the operationalization of mentalization [24], we expected to find a strong correlation between an adaptive reflective functioning (revealed by high scores at the RFQ_C scale and low scores at the RFQ_U scale) and the ability to identify, process, and express emotions.

#### Empathy

The Empathy Quotient (EQ; [20]) scale is a 60-item self-report instrument developed to assess the ability to understand other people’s thoughts and emotions and respond to them appropriately, processing the situation and experiencing—as well as showing—the same or similar feelings as the other person.

Respondents indicate their agreement with each item on a four-point Likert scale. The total score is divided into three subscales: Cognitive Empathy (the ability to infer other people’s mental and emotional states), Emotional Reactivity (proneness to react to other people’s emotions), and Social Skills (intuitive understanding of people’s emotional reactions and behaviours). Psychometrical analysis has shown that these three factors are intercorrelated, suggesting the existence of a higher-order factor of general empathy.

To avoid fatigue, we used a shorter version of the scale, consisting of 15 items and validated both in English [26] and Italian [27]. Previous psychometric analyses have shown that this 15-item version of the Empathy Quotient scale is the one with the best fit indices; the instrument has shown good reliability and a solid concurrent, convergent, and discriminant validity [26, 27].

#### Reflective functioning

The Reflective Functioning Questionnaire (RFQ; [24]) is a brief self-report instrument consisting of 8 items and developed to assess the subject’s mentalization abilities. It evaluates the capacity to understand and reflect upon our and other’s behaviours in terms of mental states (e.g., desires, intentions, beliefs, and emotions). For each item, subjects express their level of agreement on a seven-point Likert scale, ranging from 1 = “completely disagree” to 7 = “completely agree.” The total score is divided into two subscales: Certainty (RFQ_C) and Uncertainty (RFQ_U) about the mental states of self and others. RFQ_C scores are related to empathy and mindfulness abilities, while research high RFQ_U scores are associated with impulsivity, depressive affects, and self-harm tendencies [24].

The RFQ has already been validated in Italian [28], and it has shown robust psychometric properties, such as good internal consistency, construct validity, and test-retest reliability.

### Data analysis

All statistical analyses were performed using IBM SPSS Statistics 27.0 and Jamovi project software (Version 1.8.1). All data were examined for normality (skewness and kurtosis). The criterion for significance was set at *p* = 0.05 for all analyses. In addition to descriptive statistics, the following psychometric properties of the B-MAS scales were evaluated.

1. **EFA** An Exploratory Factor Analysis (EFA with Promax rotation) was performed to determine the scale structure. The number of factors was chosen according to experts’ recommendations (Kaiser-Meyer-Olkin criteria > 0.6, Bartlett’s Test of Sphericity <0.05 and plot of eigenvalues-scree-test). Through these indices, the simple structure has been explored.
2. **CFA**. Confirmatory Factor Analysis (CFA) was run on the emerged components. Standardised coefficients of ≥ 0.4 were considered acceptable [29]. Normalized mean and covariance residuals were evaluated and found acceptable. Maximum Likelihood (ML) was used as an estimation method.
3. Model fit was estimated by two absolute indices of overall model fit: root mean square error of approximation (RMSEA) and standardised root mean residual (SRMR). Additionally, one relative index of model fit was used: comparative fit index (CFI). Finally, the Tucker Lewis Index (TLI) has been computed. The acceptable thresholds for these indices were defined as RMSEA = 0.05–0.08, SRMR < 0.08, and CFI > 0.90, according to Kline’s guidelines [30] and TLI > 0.95 according to Bentler (1990).
4. **Reliability**. To assess scale reliability, we used Cronbach’s alpha. A generally accepted rule is that an α of 0.6–0.7 indicates an acceptable level of reliability, while an α of 0.8 or greater indicates an excellent level. However, values higher than 0.95 are not necessarily good since they might be an indication of redundancy [31].
5. **Convergent Validity**. Convergent validity was assessed using the constructs of empathy and reflective functioning, which are closely related to mentalized affectivity. Empathy was assessed with the Empathy Quotient (EQ) scale [26, 27], Reflective Functioning with the Reflective Functioning Questionnaire (RFQ; [24, 28]). Pearson’s r correlation coefficient was used, and only significant values were accepted as valid correlations.
6. **Effect of Demographics and Normative data**. First, we performed a multivariate analysis of variance (MANOVA) to study the effects of gender, age (years), and education (years) on the B-MAS scales. To interpret the effect size, we used eta squared values (η2) (η2 > 0.01 = small effect; η2 > 0.06 = medium effect; and η2 > 0.14 = large effect) [32]. To provide Italian normative values, we studied the effect of gender on the B-MAS scales. Gender was coded as follows: 1 = male; 2 = female; 3 = non-binary.

## Results

### Descriptive analysis of B-MAS items

The descriptive analysis of the B-MAS items is presented in Table 1.

**Table 1:** Descriptive statistics of the 12 items.

	ITEM 1	ITEM 2	ITEM 3	ITEM 4	ITEM 5	ITEM 6	ITEM 7	ITEM 8	ITEM 9	ITEM 10	ITEM 11	ITEM 12
Mean	5.52	3.93	3.97	5.48	3.64	3.72	5.75	4.12	3.90	5.67	4.44	3.05
St.dev	1.51	1.69	1.64	1.45	1.66	1.92	1.22	1.60	1.59	1.41	1.43	1.66
Minimum	1	1	1	1	1	1	2	1	1	1	1	1
Maximum	7	7	7	7	7	7	7	7	7	7	7	7
Skewness	-0.16	-0.02	0.02	-0.27	0.13	0.17	-0.15	-0.04	0.09	-0.16	-0.34	0.23
Kurtosis	0.18	0.45	-0.31	0.43	0.32	-0.21	0.30	-0.24	-0.18	0.41	-0.36	-0.26

Note: Reversed items # 5-6-10-12; st.dev. = Standard deviation.

Although there is no single way to interpret distribution shape values, our data show skewness and kurtosis values appropriate for the normal curve approximation (for details, refer to [29, 33, 34]).

### EFA—Exploratory Factor Analysis

We performed a EFA with Promax rotation on the 12 items of the B-MAS. The Kaiser-Meyer-Olkin Measure of Sampling Adequacy was .814, and the Bartlett’s Test of Sphericity was significant (*p* = <0.01). The analysis of the Scree test (Fig 1, panel B) suggested a three components solution. The three components together accounted for 61.87% of the variance. Observing the ambiguity of the factorial loading of item 3, we forced the EFA to extract a supplementary factor. Although extracting a fourth component would have explained 6% more of the variance, it would not have approximated a simple structure; therefore, we believe that the three-factor solution is the most appropriate and we have attributed item 3 to the first factor.

**Fig 1:** Panel A: EFA loadings of the three factors after Promax rotation. Values in bold show the items with the highest saturations in the factor. Panel B: Scree plot.

The rotated factor pattern (Fig 1 panel A) revealed a simple structure. All but one (item 3) of the variables have high factor loadings on only one factor and very low loadings on all the other. Furthermore, correlations among the three factors are low and nonsignificant, suggesting independence among all of them. The first extracted factor explains 31.72% of the variance; it showed strong loadings from 4 items assessing how people express and communicate their emotions to others (i.e., externalizing them). The second explains 17.29% of the variance; it showed strong loadings from items assessing people’s ability to control their emotions using cognition. The third and last factor explains 12.87% of the variance, showing loadings from 4 items evaluating a self-assessment of one’s ability to be aware of one’s own emotions. Following Greenberg and colleagues [18], we decided to maintain the same factors’ labels, namely: 1 = Expressing; 2 = Processing; 3 = Identifying.

### CFA—Confirmatory Factor Analyses

The CFA provided a statistically significant model (χ^2^ = 169; p < 0.001); as showed in Table 2, the fit statistics provided acceptable values.

**Table 2:** Fit measures.

				RMSEA 90% CI	
CFI	TLI	SRMR	RMSEA	LOWER	UPPER
0.921	0.989	0.067	0.077	0.064	0.090

Note: CFI = comparative fit index; TLI = Tucker–Lewis’s index; SRMR = standardized root mean square residual; RMSEA = root mean square error of approximation.

### Reliability

Cronbach’s alpha reliability coefficient showed excellent values for the Processing (0.799) and the Expressing (0.817) scale, and a good value for the Identifying scale (0.692).

### Convergent validity

Pearson’s r coefficients between B-MAS and EQ subscales showed significant correlations in all but one of the comparisons. As displayed in Table 3, all B-MAS correlations were positive, suggesting direct linearity with the analysed constructs. The only nonsignificant comparison was between the B-MAS Processing subscale and the EQ Emotional Reactivity subscale. Concerning Pearson’s r coefficients between B-MAS and RFQ subscales, all but one of the comparisons showed significant correlations, and among significant correlations all except one were positive. The only nonsignificant comparison was between B-MAS Expressing and RFQ Uncertainty. Moreover, RFQ Uncertainty negatively correlated with B-MAS Processing.

**Table 3:** Correlation between the three subscales of the B-MAS, the EQ scales, and RFQ scales.

		B-MAS		
		Expressing	Processing	Identifying
**EQ**	EQ Total	.301**	.251**	.349**
	Cognitive Empathy	.159**	.182**	.345**
	Emotional Reactivity	.173**	-.033	.286**
	Social Skills	.295**	.369**	.109**
**RFQ**	RFQ Certainty	.106**	.333**	.152**
	RFQ Uncertainty	.048	-.185**	.224**

Note:

* = p < .05;

** = p < 0.01;

EQ: Empathy Quotient; RFQ: Reflective Functioning Questionnaire.

### Effect of demographics and normative data

Multivariate Analyses of Variances (MANOVA) indicated a main effect of gender on the B-MAS (*Pillai trace* = 0.054; p = 0.006). Extensive investigations with univariate statistics have shown a main effect of gender on Processing (F_(2,658)_ = 3.15; *p* = 0.044) and Identifying (F_(2,658)_ = 3.9; *p* = 0.021).

LSD post-hoc suggested that males scored significantly higher than female and non-binary subjects in the Processing scale (males = 4.35, ±1.2; females = 3.77, ±1.2; non-binary = 3.55, ±1.09), while females obtained higher score than males in the Identifying scale (males = 5.4, ±1; females = 5.70, ±0.9). Two- and three-ways interactions were not significant.

Based on previous analyses showing a significant effect of gender on the B-MAS scores, normative data were elaborated separately for the three gender categories (Table 4).

**Table 4:** Italian normative data of B-MAS subscales.

		Expressing	Processing	Identifying
**Males**	Mean (St. dev)	5.79 (1.03)	4.35 (1.30)	5.40 (1.05)
	Min—Max	3.75–8.00	1.50–7.00	2.50–7.00
	25 percentile	5.00	3.50	4.75
	50 percentile	6.00	4.50	5.50
	75 percentile	6.50	5.25	6.25
**Females**	Mean (St. dev)	5.99 (1.04)	3.77 (1.23)	5.79 (0.92)
	Min—Max	3.75–8.25	1.00–6.50	3.5–7.00
	25 percentile	5.25	3.00	5.25
	50 percentile	6.00	3.77	5.75
	75 percentile	6.75	4.75	6.50
**Non-binary**	Mean (St. dev)	5.88 (1.26)	3.55 (1.09)	5.63 (1.16)
	Min—Max	3.75–8.00	1.75–5.50	3.50–7.00
	25 percentile	4.75	2.75	4.75
	50 percentile	6.00	3.50	6.00
	75 percentile	6.75	4.625	6.75

Note: St.dev. = Standard deviation.

## Discussion

### Factorial structure

The first aim of the present study was to evaluate the factorial structure of the B-MAS [18] in an Italian sample. Findings from the EFA and CFA strongly mirrored the three-factor model already proposed by Greenberg and colleagues [18], finding the same three-factors structure. However, we observed some differences in the order of those factors. In the present study, the first was Expressing, the second Processing and the third Identifying. In the original study by Greenberg and colleagues [18], instead, the first component was Processing, the second Identifying and the third Expressing. It is possible to suppose that the order of factors may be different due to the differences that exist from a linguistic and cultural point of view.

Interestingly, though, in both studies the three factors taken together accounted for around 61–62% of the variance. Despite the differences mentioned above, both the Italian and the USA structure accounted for the same proportion of the variance and showed a three-factor structure. Taken together, these results highlight both the good operationalization and robust empirical foundation of the construct, which is further corroborated by the CFA values obtained in our analysis.

Therefore, the B-MAS seems to be a promising tool for mentalized affectivity, notwithstanding its brevity. On the other hand, such brevity makes the B-MAS quite valuable for clinical and research purposes (it takes only around 5–10 minutes to complete and score it). Besides, our analyses allowed us to obtain normative data broken by gender for the Italian population: this will let clinicians and researchers to easily compare their scores with national normative values.

### Convergent validity

The B-MAS showed excellent psychometric properties. The three B-MAS subscales demonstrated good convergent validity, as they correlated with both the Empathy Quotient (EQ) and the Reflective Functioning Questionnaire (RFQ) subscales. The fact that the correlations with empathy and reflective functioning scores were significant, but rather small, seems to indicate that the construct of mentalized affectivity—thus one of its measurement tools, the B-MAS—represent, as postulated by Jurist [10], both a bridge concept and an innovative one, able to broaden the perspective on affect regulation and mentalization and to offer a quite unite point of view.

#### Correlations between mentalized affectivity and empathy scores

For what concerns empathy, almost all correlations between the three components of the B-MAS and the EQ subscales were in the expected direction. Only one correlation resulted not significant, the one between the Processing component of the B-MAS and the Emotional Reactivity subscale of the EQ, which measures the tendency to have an emotional response to others’ emotional displays or mental states (i.e., ‘I tend to get emotionally involved with a friend’s problems’). In line with Greenberg and colleagues [17], we found a negative correlation between the Processing dimensions and Emotional Reactivity scores at the EQ. This result suggests that the capacity to regulate and modulate emotions may be hindered by a strong disposition towards affective empathy, which, on the other hand, positively correlates with the ability to communicate emotions (Expressing) and “understand” them (Identifying). Both the Cognitive Empathy and the Social Skills showed positive correlations with all three components of the B-MAS. The Cognitive Empathy subscale measures the capacity to acknowledge affective states (i.e., ‘I can tell if someone is masking their true emotion’), epistemic states (i.e., ‘I find it easy to put myself in somebody else’s shoes’), and desire-based states (i.e., ‘I can easily work out what another person might want to talk about’).

Instead, the Social Skills subscale measures the individual’s proneness to use interpersonal skills and intuitive understanding abilities (i.e., ‘I often find it difficult to judge whether something is rude or polite’). The positive correlations between these dimensions indicate that mentalized affectivity is closely linked to the cognitive side of empathy (i.e., the ability to infer and understand other people’s emotions). Cognitive empathy, in turn, seems to have important similarities with the broad concept of mentalization (or reflective functioning), so much that the two expressions are sometimes used interchangeably (see, for example, [35]). Research has already shown that the mental processes related to cognitive empathy involve the activation not only of the limbic areas implicated in personally experiencing the other’s feelings but also of the neocortical networks associated with mentalization processes [36].

#### Correlations between mentalized affectivity and reflective functioning scores

Concerning the correlations between mentalized affectivity and reflective functioning, we found a positive correlation between all three components of the B-MAS (the strongest one was with Processing) and the Certainty scale of the RFQ (RFQ_C), which measures the individual’s overall mentalizing stance and abilities. As expected, we also found a negative correlation between the Processing component of the B-MAS and the Uncertainty scale of the RFQ (RFQ_U), which instead measures how much the self’s and other’s mental states tend to remain unknown, ambiguous, and/or unpredictable (i.e., ‘Sometimes I do things without really knowing why’). This result seems to confirm what was previously highlighted by other studies that found a positive correlation between the RFQ_U and alexithymia [37].

The positive correlation between Identifying and RFQ_U was, instead, an unexpected finding. The ability to identify and reflect on emotions may thus be linked with both good and lacking self-reported capacity of reflective functioning. It might be useful to remember that the Identifying dimension refers to the ability to recognize not only one’s emotions but also other people’s feelings [10]. Individuals highly attentive and vigilant for emotional stimuli (who will likely score high on the Identifying subscale) often seem to present a slight deficit, real or perceived, in the ability to correctly interpret and reflect upon self’s and other’s mental states [38]. It would be interesting to explore further the links between mentalized affectivity and reflective functioning on broader samples or using a different method for the assessment of RF, such as the clinician-rated Reflective Functioning Scale (RFS; [39]) applied to Adult Attachment Interviews (AAI; [40]) transcripts. It would also be interesting to investigate the differences between basic and higher-order emotional identification and processing [41]. As Fonagy and Luyten [42] already suggested, the mentalization deficits described above (not dissimilar to that observed in borderline personality disorder; [38]) could be the result of poor integration between a “lower”, implicit form of mentalizing, more related to affects, and a “higher” form, more related to reflective thought. Furthermore, it could be fascinating to explore how different kinds of focus (on one’s own or other’s emotions) within the Identifying dimension are linked to various forms of psychopathology.

#### Effect of demographics

Other interesting results concern the effect of gender on the B-MAS scores. In line with previous findings [17, 18], the male subjects in our sample scored higher than females and non-binary on Processing, whereas females scored higher than males on Identifying. No gender differences were found regarding the Expressing dimension. While Processing is related to the ability to distinguish between different emotions, modulating and managing them, Identifying represents a more complex component linked to autobiographical memory. The items of this scale measure how much individuals make an active effort to understand the underlying reasons of affective states and to situate their emotions within the context of their life history. It is thus not surprising that females scored higher than males on Identifying: the so-called ‘female superiority’ in terms of empathy [43, 44], emotional intelligence [45], and reflective functioning [46] is indeed a consolidated finding in the literature. There could also be a cultural factor at play: females may be more inclined to value the process of identifying emotions because they have been more encouraged to do so than males since a young age [47].

On the other hand, in line with USA findings [17, 18], we found that the (self-reported) ability to control emotions is more developed in males. Since literature shows that women score higher than men on many emotion regulation strategies [48, 49], this result is, in part, surprising. However, this finding is consistent with the cultural belief that males are more effective in suppressing and avoiding troubling emotional states, since the expression of certain feelings represents a “feminine” trait [50]. It is possible to speculate that, when self-reporting about their attitude toward emotions, male subjects may have emphasized these aspects.

Finally, non-binary respondents showed lower scores on Processing. However, their group is too small (N = 17) to perform significant comparisons. Nevertheless, literature data show that non-binary individuals are subject to many forms of discrimination and often show psychological and relational difficulties [51–53]. This may lead to problems in managing and controlling emotions, an aspect that future studies should investigate further.

#### Limitations

Our work has limitations which need to be discussed. The first one concerns the recruitment of participants, which was carried out through an online survey. Even though this procedure is being increasingly used in research, we are aware that it may lead to the exclusion of a portion of the population, specifically of individuals who have scarce access to the Internet, or who might have trouble using technology. For this reason, we consider it essential to carry out a subsequent cross-validation study involving a face-to-face administration. Nevertheless, the convergence of our results with those obtained by Greenberg and colleagues on the US population [18] corroborates, at least partially, the robustness of its geographical and cultural generalizability. Another limitation concerns the absence of a direct comparison with a clinical population, which would allow to study the discriminating efficacy of the scale and provide more useful clinical indications for psychotherapeutic practice. On the same line of reasoning, it would also be important to investigate if some variables such as having been in psychotherapy, having experienced trauma, or the presence of clinical diagnoses and other personality traits affect the scores obtained at the B-MAS. Finally, one last comment concerns the possibility that ITEM 3 could be interpreted as ambiguous (with a slightly higher load in the first factor). We believe that in a subsequent cross-validation study this hypothetical ambiguity can be clarified.

## Conclusion

Mentalized affectivity is emerging as a relevant construct in literature: it encompasses different aspects of emotion regulation (such as the ability to process, express, and identify emotions), and it could pave the way to interesting clinical and theoretical findings. As already mentioned, the brevity and ease of administration of the B-MAS make it particularly valuable both in clinical and research contexts. The results of our study highlight how this instrument represents a promising tool. Specifically, we found an adequate replication of the original three-factor solution, yielding three subscales with excellent scale reliability, as well as convergent validity with other related constructs. Finally, although it is crucial to cross-validate the results of our study, the normative data provided in the paper provide a first benchmark for the comparison of the scores obtained by different samples (e.g., individuals with a clinical diagnosis, individuals who have experiences various forms of trauma, and so on) both in clinical and research contexts.

## Supporting information

S1 Data (SAV)
